# Quantitative Evaluation of Vocabulary Emotional Color in Language Teaching

**DOI:** 10.1155/2022/5203122

**Published:** 2022-04-13

**Authors:** Zhong Caihong

**Affiliations:** ^1^The University International College, Macau University of Science and Technology, Macao 999078, China; ^2^The International College, Sichuan International Studies University, Chongqing 400031, China

## Abstract

**Objective:**

In real communication, the context is complex and changeable and the color and meaning of some words will wander in the context. The development and changes of words are more complex and multidimensional than before. Compared with the rational meaning of words, the color meaning of words can better reflect the psychological mode and way of thinking of the Han nationality but it is difficult for foreign learners to accurately grasp and misunderstandings often occur. In order to solve this problem, it is necessary to summarize and explain the words whose color meanings are easily shifted, so as to help the students accurately grasp the color meanings of the words and better help Chinese learners to realize the communicative function of the language.

**Method:**

This paper takes the scope of emotional words as the starting point and proposes that emotional words are words with emotional colors. The four aspects of whether words belong to emotional words define the concept of emotional words and introduce the specific methods of judging and extracting emotional words from the two aspects of dictionary definition and word collocation. This paper takes foreign students whose native language is English as the research object, through questionnaire survey and corpus analysis, to investigate the use of foreign students' emotional colors and to explore the influence of native language factors on emotional color acquisition. Based on the research of modern Chinese ontology and the existing research results in the field of teaching Chinese as a foreign language, this paper takes the theory of interlanguage and transfer theory as the theoretical basis and mainly uses the methods of comparative analysis and error analysis to try to find out the relationship between emotional color teaching and acquisition.

**Results:**

/*Discussion*. The basic pattern and quantity distribution of lexical emotion correction for beginners, intermediate, and advanced learners of Chinese as a second language were analyzed, and the restrictive factors and characteristics were explained. Similarities and differences and the rationale behind them were explored. In the process of international Chinese teaching, teachers mostly pay attention to the rational meaning of words, while ignoring the teaching of the emotional meaning of words. The lack of vocabulary emotion and meaning teaching is prone to errors in students' understanding and use. With the increase of the vocabulary of intermediate and advanced learners, many words with similar colors and meanings appear, which brings a lot of difficulties for students to distinguish between synonyms. If the use of words with emotional meanings is not accurate, it is easy to cause communication barriers.

## 1. Introduction

Language is the most important communication tool for human beings, and its status and role in communication activities are self-evident [1]. Chinese itself is composed of many elements such as pronunciation, Chinese characters, vocabulary, semantics, and grammar, and vocabulary is one of the elements of language. It is the bearer of pronunciation and semantics, and grammatical rules are also reflected by the combination of words. It is its ability to form words into sentences and the function of conveying information that make it the most powerful participant in the process of language communication [2]. In other words, without vocabulary, communication activities cannot be carried out.

It is precisely because of the important position occupied by vocabulary in language communication that vocabulary teaching should be a part that cannot be ignored in the process of teaching Chinese as a foreign language [3]. Many experts and scholars attach great importance to vocabulary teaching in teaching Chinese as a foreign language [4–6]. They advocated that “vocabulary teaching should be the center” in teaching Chinese as a foreign language [7]. For learners who use Chinese as a second language, vocabulary learning and accumulation are the basis for enhancing their communicative ability. Only when they have enough vocabulary can they have the cornerstone of word choice and sentence construction. However, it is necessary to know how to choose suitable words in different communication situations to express the meaning with expressions, so as to have a targeted, natural, and appropriate way of speech communication [8]. The additional meaning of word meaning is also called word color meaning, which mainly includes emotional color, image color, and stylistic color. The emotional color of words generally refers to the positive and negative meanings of words, which can express the subjective emotions and attitudes of the speaker. The image color of words often enables readers to form a vivid understanding of things through words. For learners who use Chinese as a second language, they can grasp the basic meaning of words, that is, the rational meaning of words, through the interpretation of words [9].

In the past research, the research on the rational meaning of words has always been the focus and fruitful results have been achieved [10, 11]. In a word, as an important part of the meaning of word color, word style color has received relatively insufficient attention, so it is necessary to conduct a special study on word style color.

In the teaching of Chinese vocabulary as a foreign language, the identification and analysis of synonyms have always been a difficult point in the teaching process [12]. For learners whose native language is not Chinese, the rational meaning annotation of the dictionary is an important way for students to understand the meaning of words [13]. There are a large number of synonyms, and there is little difference in the rational sense. Even when annotating the meaning of a word, a common word with low difficulty is often used to explain another word with the same or similar meaning [14].

In addition to the teaching of vocabulary meaning, the additional meaning of words, that is, color meaning, should also be paid attention to in vocabulary teaching [15]. In addition to understanding the rational meaning of words, students should also understand when to use words in which style of language to meet the requirements. When words are basically the same in concept expression, in order to distinguish their nuances in practical application, it is necessary to start from the emotional color and style color of words [16]. The labeling is mostly used for derogatory meanings and mostly used for commendatory meanings. The specific use of a word should consider factors such as occasion, participants, and communicative purposes. This requires a clear understanding and ability to distinguish the style and color of the word [17, 18].

The purpose of this paper is to sort out words whose color meanings are prone to shift. Through the multifaceted analysis of various use cases, we can make everyone have more understanding and cognition of the problem of vocabulary color meaning wandering and hope that this can help Chinese learning. Students will have an in-depth understanding of the characteristics of Chinese communication and use Chinese appropriately.

## 2. Methods

### 2.1. Definition of the Color of Emotional Words

Words are divided into monosemous words and polysemy words; so, to discuss the emotional color of words, it is necessary to gradually classify and discuss specific meanings. From the point of view of the meanings of emotional meanings, we can divide emotional words into two cases, namely, emotional words on all meanings and emotional words on partial meanings. The emotional color on all senses means that each sense of a word has emotional color, which includes two situations: one is that a single sense has only one sense and this sense has emotional color and the other is that each sense of a polysemy has emotion. Emotional words on partial senses are for polysemy, which means that if a polysemy does not have every sense with emotion but only one or several senses have emotion, then, we think that it belongs to partial sense. When discussing emotional words, it is necessary to make specific analysis based on the specific meanings of the words and it is not possible to generalize these two situations in general.

In addition, it should be pointed out that there are two kinds of components of vocabulary; one is word, that is, the smallest unit of sentence making that can be used independently in the language with the combination of sound and meaning; the other is a fixed structure equivalent to the function of words. When we describe emotional words, we do not make a strict distinction between the usage of “word” and “language,” both of which are lexical units of emotional meaning, so we use the term “emotional words.”

For words expressing feelings such as “like,” “sad,” “pain,” and “anger”, their rational meaning is itself a positive or negative evaluation of objective things. Emotional words should refer to those words whose rational meaning does not contain praise or criticism but have a tendency to praise or criticize in terms of meaning. Therefore, the two are fundamentally different and cannot be confused.

This paper believes that emotional words and words expressing feelings are essentially different and should be treated differently. Words expressing feelings do not belong to the research object of this paper.

The emotional meanings of the emotional words that we say should be relatively stable, independent of the temporary context or context in which the words appear, and the meaning content of which can be independently analyzed in the meaning of the words. Therefore, emotional words in this rhetorical sense are not within the scope of our discussion.

### 2.2. The Extraction Method of Emotional Words

The collection of such words in the special dictionary of emotional words allows readers, especially international students, to have a relatively clear standard in the judgment of the emotional meaning of words. In addition, the definitions and example sentences in the dictionary also show readers a complete and accurate picture, so that it can correctly understand and use emotional words.

Emotional words are generally divided into positive words, derogatory words, and neutral words, which is also called the “rule of thirds.” There are also some scholars who believe that this trichotomy is not enough to express the vastly different emotions of human beings, so they advocate that emotional words should be divided more carefully on the basis of the trichotomy [4, 7]. For example, related scholars have classified emotional words from two perspectives [11]. One is to divide emotional words into fourteen types in terms of nature; the other is to divide emotional words into two types in terms of specific content.

Between the opposite ends, there is an intermediate expression where the two sides do not rely on each other, which is a general attitude. Each attitude color shows its peculiarity because of its comparison with ordinary attitudes. Naturally, if a word is ordinary or neutral in attitude, it does not have any attitude color.

We believe that neutral words still have emotional colors. It is just that the expression of its emotional color is not as obvious as positive and derogatory words. Therefore, this article focuses on the emotional color of positive words and derogatory words and does not discuss too much about neutral words.  Figure 1 shows the mode of lexical emotion correction of Chinese as a second language learner.

Chinese scholars have also conducted in-depth research on the method of examining the emotional color of words through word collocation. This method is mainly used to discuss the emotional color choice of verbs to objects. There is a semantically cooccurrence-constrained relationship between verbs and objects, that is to say, the object of a verb must meet the semantic characteristics of the verb and must be something specified or required by the semantics of the verb. It must be something that its object can participate in.

By observing the context in which these words appear in the corpus, it can be seen that some emotional words that are not clearly marked in the dictionary are often affected by the context because they often appear in the context of praise or derogation. Through such analysis, these words can also be counted as emotional words.

### 2.3. Survey Objects

Since the mastery of emotional words is affected by Chinese proficiency, the research object is limited to international students with advanced Chinese proficiency. The survey objects selected in this paper are international students from the School of International Education and International Exchange. This paper selects foreign students whose native language is English as the survey objects of this paper, a total of 41 people. The Chinese proficiency of these international students is above level 5, and some have reached level 7. The visualization of the basic situation of the survey objects is shown in Figure 2.

### 2.4. Questionnaire Design

This questionnaire mainly investigates and researches three questions: (1) to investigate the understanding and use of emotional colors by international students in English-speaking countries and to obtain real corpus of emotional colors used by international students to prepare for the analysis of errors in the following sections, (2) by arranging the corpus, summarizing the characteristics of interlanguage, to explore the problems in the process of emotional color acquisition and determine the focus and difficulty of emotional color teaching, and (3) the questionnaire will further explore the possible influence of the English background on emotional color acquisition.

In order to ensure the reliability and validity of the questionnaire, before the formal investigation, we first carried out prediction and evaluation in the senior class of the School of International Exchange and made appropriate adjustments and modifications to the questionnaire according to the pre-examination. The revised questionnaire was then distributed to the test subjects, and they were required to complete it independently within 100 minutes. During this period, they were not allowed to read dictionaries and other materials and they were not allowed to ask others. We have made a specific explanation to the students before the questionnaire is carried out. This is not an exam, but to complete a survey to eliminate students' nervousness and ensure the quality of the questionnaire. Most of the questionnaires were completed in class under the supervision of teachers, and a small number of students handed it in after class.

The questionnaire is mainly composed of four parts: multiple choice questions, true/false questions, word choice, reading comprehension, a total of 50 questions, 2 points for each question, and a total of 100 points. The design of the questions is shown in Table 1.

When compiling the topic, this paper firstly selects emotional words as corpus from the Outline of Chinese Proficiency Vocabulary and Chinese Character Grades and Chinese textbooks based on the concept of emotional color, combined with my own teaching practice; the words examined are the frequency comparison of international students. This paper also refers to the works of “Research and Teaching of Chinese Synonyms,” “Research on Teaching and Acquisition of Chinese Vocabulary as a Foreign Language,” “Analysis of Commonly Used Chinese Synonyms,” “Dictionary of Praise and Negative Meanings of Modern Chinese Words,” and so on. All the vocabulary in the questionnaire is included in the “Chinese Proficiency Vocabulary and Chinese Character Grade Outline.” The design of the questions and options basically does not have uncommon words or supersyllabus words, so as to ensure that international students can understand the meaning of the questions.

## 3. Results

### 3.1. Vocabulary Classroom Teaching Results

The classroom observation involves a total of 153 adjectives, including 25 for A-level vocabulary, 48 for B-level vocabulary, 52 for C-level vocabulary, and 28 for D-level vocabulary.

Out of 153 adjectives, 107 adjectives are presented using the vocabulary. Teachers use the textbook vocabulary list, directly display or write the vocabulary on the blackboard, and then read the interpretation. 17 adjectives are presented using perceptual presentation, and vocabulary is presented using cards or multimedia pictures. 10 semantic fields are presented, and the target words are presented in semantically related chunks.

The vocabulary presentation method is relatively simple, and 70% of the adjectives are presented in the vocabulary list. At this stage, the classroom atmosphere is relatively dull and the students and teachers are not very enthusiastic. If the learning effect is not good and the teacher finishes reading, when students are asked to read aloud alone, the error rate is high, such as wrong intonation, wrong polyphonic words, or wrong recognition of Chinese characters. The quantitative assessment of the importance of adjective presentation is shown in Figure 3.

In the adjective presentation stage, occasionally, some adjectives can be presented with the help of example sentences in the text. For example, “these eggs are too old to be fresh” and “although he is still a child, his mind is very mature.” These can show the positive color of the new words. But most of the text examples are not typical enough to reflect the emotional meaning of adjectives. For example, “it is bad luck on the road.” The example sentences show no adjective emotion at all. 67% of the adjectives are presented in the vocabulary, and the new words are not translated into English, and the example sentences do not clearly show the emotional meaning to the students.

12.4% of adjectives are presented in context, and contextual presentation is the easiest way to present the emotional meaning of adjectives, but teachers use less and the number of new words in “Boya Chinese” is relatively large (Boya Chinese: Pre-Intermediate Acceleration I). Each lesson has an average of 31 new words, and each lesson of “Boya Chinese: Pre-Intermediate Accelerated II” has an average of 45 new words, and the presentation time of new words is limited.

There is a lack of emotional meaning presentation, and some new words are misleading students when they are presented, and they do not show the correct emotional meaning. The thirteenth lesson of “Boya Chinese: Pre-Intermediate Accelerated I” is the word “active.” The teacher designed a restaurant scene where the waiter came to help when there was no customer's call. The teacher used this to present the word “active,” but the teacher did not express his affirmation or denial of this behavior. Some students would understand that “active” was a derogatory color. In the interpretation stage of the emotional meaning of adjectives, local teachers recorded 153 adjectives for teaching when explaining vocabulary, 70 words were taught by the translation method, and the rest of words were interpreted by the comparison method, situational method, and direct method. The translation method is the most used interpretation method.

The interpretation of the 20 adjectives is a contrastive method, with synonyms or antonyms for interpretation. For example; “sweetness” in lesson 4 of “Boya Chinese: Pre-Intermediate Accelerated II” is interpreted as “very happy.” In the use of direct methods, such as the adjective “elegant” in lesson 7 of “Developing Chinese Intermediate Spoken Language II”, the teacher directly uses pictures to explain.

There are 6–8 class hours of comprehensive classes a week, using the textbook “Boya Chinese: Pre-Intermediate Acceleration”, and the teacher usually spends one class hour (50 minutes) to explain new words in one class. It takes an average of about one minute to teach a word, and the interpretation is mainly based on the teacher's translation method. A total of 48 adjective definitions were collected, of which 39 words used the translation method. Other methods are occasionally used.

In the interpretation of emotional meaning, there are several situations such as correct interpretation, deviation, and wrong interpretation. For words such as “trouble, beautiful, and comfortable” in grade A vocabulary, only using the translation method will not cause errors in emotional meaning. The two languages have common emotional meanings. Once the teacher interprets the rational meaning, the students will be able to grasp the emotional meaning and express them correctly in sentence-making practice.

The B-level word “long history” is translated as a long time, losing the positive meaning of the word “long history.” Students make sentences, point to the dilapidated classroom and say “this classroom is very old,” using “long” as a derogatory term. Sometimes, misunderstanding is caused by the teacher's atypical and inappropriate examples. For example, “hard-working,” the teacher gave an example: “Chinese people are very hard-working, they like to work very much.” With such an explanation, students do not think “hardworking” is a positive word or even a derogatory word. They think that nonstop work is like a machine. When the teacher explained the vocabulary, the example sentences were very random and subjective and failed to accurately show the emotional meaning of the adjectives.

For some words, after the teacher's interpretation, the students did not understand and grasp the emotional meaning. For example, the word “elegance” is shown by the teacher with pictures and there is no cultural background introduction or social aesthetic explanation, so that students think that “elegance” describes a certain type of painting style.  Figure 4 shows the statistics of the emotional meaning of adjectives.

### 3.2. Quantitative Distribution and Preference Analysis of Emotional Color Correction of Vocabulary in Primary Classrooms

Through the examination and analysis of the collected corpus, we obtained the frequency and frequency of vocabulary emotion correction used by elementary Chinese second language learners, as shown in Table 2.

After research, we found that among the elementary Chinese second language learners' vocabulary and emotional color correction, the number of other exercises was the largest, followed by self-initiated self-learning and self-initiated self-learning and the number of self-initiated other exercises was the least. The language level is limited, and there are certain problems in pronunciation, vocabulary, syntax, etc., and these problems have the influence of the “negative transfer” of the mother tongue. Elementary Chinese as a second language learner has difficulty noticing the problems in speech output and relies on teachers to initiate corrections. If the problems in the learners' speech are outside their “proximal development zone”, even if the teacher initiates corrections, the learners will not be able to do so. Therefore, Chinese second language teachers tend to make direct corrections from other teachers. This direct correction can enable learners to quickly and accurately notice their own language problems, thereby increasing their comprehensible input.

Comprehensible input is a necessary condition for second language acquisition, and sufficient intelligible input is the only way to acquire language knowledge. Although overemphasizing the role of external language input and ignoring the learner's own subjective initiative, we have to admit that a large amount of rich comprehensible input is a prerequisite for learners to acquire language knowledge. For second language learners, sufficient intelligible output cannot be achieved without sufficient intelligible input. Therefore, in the corpus that we collected, there were a total of 130 cases of teacher-other-initiated corrections by others, accounting for 39% of the total number of corrections at the elementary level, and the frequency reached statistical significance.

### 3.3. Quantitative Distribution and Preference Analysis of Emotional Color Correction of Vocabulary in Intermediate Classrooms

Through the examination and analysis of the collected corpus, we obtained the frequency and frequency of vocabulary emotion correction of intermediate Chinese second language learners, as shown in Table 3.

After statistics and analysis, we found that in the revision of the intermediate level, self-initiated self-cultivation ranks first and other-initiated self-cultivation ranks second, followed by self-initiated self-cultivation and finally self-initiated self-cultivation. This shows that the language ability and level of Chinese second language learners have been improved to a certain extent at this stage, they no longer rely on others to initiate corrections but can carry out a certain amount of self-initiated self-study, and their speech output is closer to the native language. However, there is still a certain gap. Therefore, the correction initiated by the Chinese second language teacher is mainly based on the teacher's own correction, which shows that the language level of the learner has yet to be developed and also reminds the Chinese second language teacher to think about which correction method is easier to start.

### 3.4. Quantitative Distribution and Preference Analysis of Emotional Color Correction of Advanced Classroom Vocabulary

Through the examination and analysis of the collected corpus, we obtained the frequency and frequency of vocabulary emotional color correction used by advanced Chinese as a second language learners, as shown in Table 4.

In the lexical emotion correction of advanced second language learners of Chinese, our corpus statistics show that the order of correction types is self-initiated self-study, other-initiated self-repair, other-initiated other-repair, self-initiated, and other repair. The language level of Chinese second language learners at the advanced stage is basically close to the language expression level of native speakers, and their classroom communicative activities are more similar to the communication between native speakers and native speakers. Therefore, the proportion of self-initiated self-study is significantly higher than that of Taekwondo, which ranks first, and with the enhancement of his language ability, the frequency of Taekwondo's self-study increases and the frequency increases significantly. To make the verbal communication activities in the classroom proceed more smoothly, the focus of its revision has gradually shifted from the language form to the transmission of communicative information and the exchange of meaning.

### 3.5. Analysis of Characteristics and Influencing Factors of Quantitative Evaluation

Through the statistics and analysis of the collected corpus, we have obtained four characteristics of Chinese as a second language learner's lexical emotion correction:

First, Chinese as a second language learner's lexical and emotional color correction in each level shows a situation that he is more enlightened than self-enlightened and self-study is more than others. We believe that this feature is completely consistent with the characteristics of the Chinese second language classroom itself. The target of Chinese second language teaching is language learners who have not fully acquired Chinese, although their language output level will increase with the improvement of their language ability. Second language Chinese teachers will consciously promote the development of learners' interlanguage through different strategies according to the learners' language ability, reduce the “negative transfer” of the mother tongue, and continuously improve the self-monitoring awareness of the interlanguage, so as to ultimately improve the learners' language level, communicative competence and communication level. The ultimate realization of this goal depends on the learner getting enough intelligible input from the language teacher; this intelligible input is controlled by the language teacher. No matter what the level of language development of learners in Chinese second language classrooms, there must be more enlightenment from others than from self-study and more from self-study than from others.

Second, in the revision of Chinese as a second language learner's lexical emotion, the ratio of self-initiated self-study to other-initiated study increased with the improvement of Chinese as a second language learner's language proficiency. The success of second language learning can be measured by the ratio of self-initiated self-study to other students' self-study.

Third, in the correction of vocabulary and emotion color of Chinese as a second language learner at each level, self-enlightenment and other revisions are always the last and the number is extremely limited. We believe that this is related to the lack of ability of Chinese second language learners to implement a certain speech act, specifically the lack of language ability of the learner to express the psychological state of hope or need. It shows that the language communication ability of Chinese second language learners needs to be improved.

Fourth, Chinese as a second language learner's vocabulary emotion correction is generally in line with the self-initiated self-correction priority mode proposed by SJS, but as an institutional conversation correction in the classroom, it has some characteristics that are different from general conversation correction.  Figure 5 shows the influence of the types of vocabulary emotion color correction features on Chinese language teaching for Chinese second language learners.

## 4. Discussion

### 4.1. Lexical Color Meaning Ontology

It is a well-established fact in linguistics that words have color meanings [19, 20]. However, the color meaning of vocabulary is a pure land that has not yet been opened up in the subject of Chinese ontology. Although many scholars have studied it, in general, the research results of color meaning of vocabulary are not fruitful [21].

In terms of emotional color of words, academic circles pay more attention to the definition and classification of emotional color of words and have achieved more results in this aspect [22, 23]. The academic community mostly uses positive words, derogatory words, and neutral words to classify the emotional color of words. However, as mentioned above, this classification is not suitable for the classification of the emotional color of adjectives. In addition to the definition and classification, linguistics has also touched on the historical evolution of the emotional color of words and the changes in their dynamic use, but overall, there are not many achievements.

In terms of the connotation and classification of the stylistic color research of words, the views on the connotation of stylistic color are basically the same: some words are often used in a certain style and these words have some stylistic color. In terms of classification, the now accepted classification is to divide it into spoken, written, and common words. The research on Chinese style ontology pays more attention to the general analysis and description of style characteristics, and the research on the relationship between style and vocabulary, grammatical structure, and style acquisition is slightly insufficient [13, 17].

In terms of the image color of words, some scholars study the image color of words from the relationship between image meaning and rational meaning [24, 25]; some scholars study the image color of words from the perspective of rhetoric [26]; some scholars study the characteristics of word formation of words with image color [27]; some scholars study the image color of words from the perspective of cognitive mechanism and other psychology [28]. But in general, there is no convincing statement in the academic circles about the connotation, classification, and pragmatic function of the image color of words.

To sum up, the ontology research on the color meaning of words is still a new discipline [29]. Even for the classification of the color meaning of words, there is no unified view in linguistics, not to mention a series of studies on its subordinate emotional, stylistic, and figurative colors. The lack of ontology research directly leads to the difficulty of teaching foreign Chinese vocabulary color and meaning as water without source and tree without roots.

### 4.2. Problems with Teachers in the Teaching Process

Cultivating students' relevant language sense is gradually mastered in a step-by-step process. However, at present, in the field of Chinese as a foreign language, the teaching of color meaning of vocabulary has not received much attention. Relevant theoretical works are quite scarce [10, 23]. Whether in the syllabus or in the textbooks, the requirements and knowledge points for the knowledge of vocabulary color and meaning are basically not covered [12, 19]. This leaves teachers with no basis for teaching, unable to correctly teach students the correct knowledge, and no teaching direction for the teaching of vocabulary, color, and meaning. In this way, many teachers have weakened their awareness of the meaning of vocabulary color, which leads to the lack of targeted teaching for the meaning of vocabulary color in specific teaching. Students' knowledge input comes from teachers. If teachers do not give students relevant knowledge input, students lack relevant knowledge and errors will naturally occur.

Although most foreign Chinese teachers believe that the color meaning of vocabulary is very important, it is necessary to teach it as a knowledge point in the classroom but the syllabus and teaching materials do not contain relevant knowledge points, so it is impossible to start [30]. Although some teachers study it, there are only a few, and the situation cannot be changed for the time being.

In addition, this paper believes that teachers also have some problems in teaching. The professors in the teacher's classroom are too reliant on the textbook. It is true that textbooks are the most important teaching books but language learning and mastery, especially vocabulary, color, and meaning, require a large amount of language material input in order to be internalized into one's own knowledge reserve. However, teachers are not sufficiently prepared for the relevant knowledge points and students are not in place to master the color and meaning of words, which will also lead to the occurrence of errors.

In the analysis of synonyms, if the teacher cannot accurately explain the difference between the two words, the students are very likely to generalize one word to another word, causing errors. For example, “popular” and “dominant,” “popular” has a strong spoken language color. If teachers only focus on explaining the rational meaning of “popular” and ignore its style color, it is easy to use “popular” in written language.

Teachers' lack of knowledge, not only knowledge of Chinese but also knowledge of foreign students' mother tongue. The research objects of this paper are foreign students whose native language is English, and the translations corresponding to the new words in the two sets of textbooks used are English translations. Although the rational meanings of the two are very similar, “in most cases, due to the difference in the additional colors, they cannot be directly translated.” If the teacher's understanding of the English translation words is not comprehensive enough but simply comprehends the two correspondingly when teaching, it will also cause the corresponding negative transfer of the mother tongue.

In addition, based on my own experience, consulting other teachers of Chinese as a foreign language and consulting relevant materials, we found that in teaching Chinese as a foreign language, teachers have very low requirements for students' recitation and generally do not require them. However, knowledge points need a lot of repeated practice to learn. Although it is too mechanized, this paper believes that a considerable degree of recitation is needed, which will help students better remember relevant knowledge points. In future practice or communication, if you can find it in the memory retained in the brain and apply it again, in the long run, you will be able to better grasp the relevant knowledge.

For knowledge points such as color meanings of adjectives, the research on Chinese ontology is not comprehensive and in depth [26]. Even if teachers themselves pay attention to color meanings, they have no way to start with them and the quality of teaching is even more difficult to guarantee. The lack of understanding of knowledge leads to inappropriate explanations in teaching, which can easily lead to negative transfer of the target language and cause errors.

Some errors are caused by misleading or neglected explanations by teachers. “Learning transfer” is a concept in psychology, which refers to the influence of acquired knowledge, skills, and even learning methods and attitudes on learning new knowledge and skills.

The target language will have an impact on the process of foreign students learning Chinese, and the impact can be divided into positive and negative. When the native language has a positive impact on Chinese acquisition, the transfer is called positive transfer; when the native language has a negative impact on Chinese acquisition, it is called negative transfer.

### 4.3. Problems with Students in the Teaching Process

Chinese learners who have entered the intermediate and advanced stages have already mastered a certain basic knowledge of Chinese and can use Chinese to complete basic communication tasks in life, study, and work [31]. In order to achieve a higher level of Chinese, in addition to mastering more vocabulary and grammatical knowledge points, students are also required to have a higher level of Chinese communication skills. Words are the smallest grammatical unit. To communicate properly, you must understand them correctly. However, the lack of ontology research has made the teaching of Chinese as a foreign language a blind spot for the teaching of vocabulary color meaning, which makes students lack of ideological understanding of vocabulary color meaning and lack of related vocabulary color meaning awareness. Their understanding of vocabulary mastery is that as long as they master the rational meaning of the vocabulary, they can use the word to make sentences even if they have basically mastered the vocabulary [32].

The reason why the research on lexical color meaning ontology is blank is that the lexical color meaning itself is abstract, intricate, and elusive. “Vocabulary itself is an open system, almost every word has its own personality, and there are not many commonalities, which is not convenient for systematic teaching [33].” Therefore, the color meanings of words are difficult to understand. Chinese-speaking learners can still rely on long-term premonitions to identify and analyze the color meanings of words. However, international students lack such innate premonitions. Not enough, the acquisition of vocabulary color and meaning is more difficult for them, so they will have a fear of related knowledge and use avoidance strategies in use. Without the internalization, practice, and use of relevant knowledge, the acquisition of vocabulary color and meaning will be even more insufficient. Such a vicious circle will further lead to a series of biases.

The identification and analysis of synonyms are a headache for international students. They have basically the same rational meaning, but words with different collocations and usages will cause confusion and errors. After learning a word and understanding its rational meaning, students use the word widely, ignoring whether it conforms to the context, whether the collocation is appropriate, whether there are errors in usage, etc., resulting in errors. For example, “calm” and “quiet,” international students think that “calm” also means “quiet,” which results in the generalized use of the word “calm.”

There is also a common error in the analysis of synonyms, which is the generalization of monosyllabic words into various related disyllabic words, resulting in inappropriate language. There are many relevant examples of the above bias, such as using “bitter” as “painful” and “honey” as “sweet.” Because these words have common morphemes in morphological form, the semantics are related or relatively similar, which makes students indistinguishable in the initial use, resulting in the generalized use of monosyllabic words.

Students' lack of understanding of vocabulary is not only because there is a lack of understanding of the words themselves but also because the translation and interpretation of the words in the textbooks are not in place. Due to various reasons such as cultural background, cultural factors are implicit in the vocabulary system, because the composition of the vocabulary system of any language is affected by social conditions, religious beliefs, customs, values, ways of thinking, and aesthetic taste [34]. There are various differences between two different languages. Except for some purely objective directional words, it is rare to find two completely corresponding words in the two languages. However, when students learn vocabulary, they often only pay attention to the rational meaning of vocabulary, especially for unfamiliar words; international students will simply correspond to them in their native language and apply the context, usage, and collocation of native language words to Chinese words by themselves.

## 5. Conclusion

Vocabulary teaching has always been a difficult point in Chinese teaching, and vocabulary teaching has received more and more attention. However, adjective teaching attaches great importance to the rational meaning and the emotional meaning of the vocabulary is not enough. Therefore, in practical teaching, the phenomenon of learners' use of emotional meaning is often inappropriate. The large number of synonyms in adjectives and the rich emotional meaning of adjectives have brought some difficulties to students. In the revision of Chinese as a second language learner's vocabulary emotion color, the ratio of self-initiated self-study to other-initiated study increased with the improvement of the language level of Chinese second-language learners, indicating that the language ability of the learners is getting closer and closer to the native language. Therefore, the language communication activities in the classroom are also carried out more smoothly with the improvement of the second language learners' verbal communication ability and the teaching objectives are easier to achieve. Complexity has also increased, making classroom interactions between teachers and students, as well as between students, more efficient. Through the research on the lexical and emotional color correction of Chinese as second language learners, it is suggested that our Chinese second language teachers should strive to combine scaffolding teaching with the theory of conversation correction and build “scaffolding” for learners in classroom interaction. The establishment of a sexual framework enables learners to maximize their existing language abilities within the “zone of proximal development” and then internalizes them into new inherent knowledge and finally realizes the learners' autonomous learning after the “scaffolding” is removed.

## Figures and Tables

**Figure 1:** The mode of vocabulary emotion correction of Chinese as second language learners.

**Figure 2:** Visualization of the basic situation of the surveyed subjects. (a) Chinese proficiency; (b) age distribution; (c) gender ratio.

**Figure 3:** Quantitative assessment of the importance of adjective presentation.

**Figure 4:** Statistics of the emotional meaning of adjectives.

**Figure 5:** The influence of the types of vocabulary emotion color correction features on language teaching.

**Table 1:** Questionnaire design.

Question type	Intention to investigate	Quantity
Choice of words fill in the blank	To examine students' understanding and use of emotional colors	7
Reading comprehension	To examine the ability to understand the emotional coloration at the pragmatic level	14
Multiple choice	Select words with different emotional colors to set up options to test whether international students can use them correctly	11
True or false	Test whether students can make correct judgments on the emotional color of words	18

**Table 2:** Vocabulary emotion correction types and frequency of use by elementary Chinese as second language learners.

Correction type	Self-study	Self-initiated	Self-study by others	Initiation and revision	Total
Frequency of use	131	9	73	152	365
Frequency	38	3	21	48	110
Sequence	2	4	3	1	

**Table 3:** Vocabulary emotion correction types and frequency of use by intermediate Chinese as second language learners.

Correction type	Self-study	Self-initiated	Self-study by others	Initiation and revision	Total
Frequency of use	124	2	43	102	271
Frequency	52	1	18	42	113
Sequence	1	4	3	2	

**Table 4:** Vocabulary emotion color correction types and frequency of use by advanced Chinese as second language learners.

Correction type	Self-study	Self-initiated	Self-study by others	Initiation and revision	Total
Frequency of use	93	3	87	69	252
Frequency	40	2	36	30	108
Sequence	1	4	2	3	

## Data Availability

The data used to support the findings of this study are available from the corresponding author upon request.
